The article "The Prediction of a 3-Protein-Based Model on the Prognosis of Head and Neck Squamous Cell Carcinoma" was published in 2022. Journal: Comput Math Methods Med.

# The Prediction of a 3-Protein-Based Model on the Prognosis of Head and Neck Squamous Cell Carcinoma

**DOI:** 10.1155/2022/2161122

**Published:** 2022-06-17

**Authors:** Xiaoting Chen, Kaiyi Wong, Yixuan Li, Zhong Guan

**Affiliations:** Department of Otolaryngology, Sun Yat-sen Memorial Hospital, Sun Yat-sen University, Guangzhou, China

## Abstract

**Background:**

Head and neck squamous cell carcinoma (HNSCC) is one of the commonest malignant tumors. Using high-throughput genomic methods, RNA-based diagnostic and prognostic models for HNSCC with potential clinical value have been developed. However, the clinical utility and reproducibility of these models are uncertain. Because the complex regulatory processes occurring after mRNA is transcribed, the abundance of proteins in a cell can never be fully predicted or explained by their corresponding mRNA expression. We aimed to assume and verify a novel protein signature for checking the HNSCC patients' prognosis.

**Methods:**

The functional proteomic data of 332 HNSCC cases were collected from The Cancer Proteome Atlas (TCPA), and the related follow-up and clinical data were acquired from The Cancer Genome Atlas (TCGA). This study adopted multivariate and univariate Cox regression analysis, Akaike Information Criterion, receiver operating characteristic (ROC) analysis, and Kaplan-Meier method.

**Results:**

Patients' clinical features in both sets were comparable (all, *P* > 0.05). The area under the ROC curve (AUC) for the 3-protein signature (X4EBP1_pT37T46, HER3_pY1289, and NF2) in the test set was 0.655 and in the combined cohort (all 332 patients combined) was 0.699. In addition, the 3-protein signature exhibited better predictive value for the survival of HNSCC patients as in comparison with conventional clinical factors like age, gender, tumor stage, and smoking history (TNM stage).

**Conclusion:**

The 3-protein signature developed in this study exhibits good performance in predicting the overall survival of with HNSCC patients. The 3-protein signature exhibited better predictive value for survival than conventional clinical factors just like gender, TNM stage, smoking history, and age.

## 1. Introduction

Head and neck squamous cell carcinoma (HNSCC) is a malignancy originating from the oropharynx, hypopharynx, oral cavity, and larynx. More than 550,000 persons worldwide are diagnosed with HNSCC annually, resulting in 380,000 deaths [1]. Epidemiological studies have indicated HNSCC's incidence is growing, and the 5-year survival rate is <50% despite advances in treatments such as surgery, radiation therapy, and chemotherapy [2–5]. The survival rate is <1 year in locally advanced HNSCC patients who develop metastases or relapse [6]. Alcohol consumption, human papillomavirus (HPV) infection, and smoking are related to the occurrence, progression, and prognosis of HNSCC [7]. However, the reliability of these risk factors is unclear [8]. HNSCC associated with tobacco use and HPV have been shown to have different molecular signatures, complicating the use of molecular techniques to predict survival and develop targeted treatments [9]. Because of the molecular heterogeneity and etiological complexity of HNSCC, it is difficult to determine novel biomarkers that can help prognosis prediction and therapy guidance [8, 10]. Using high-throughput genomic methods, RNA-based models with potential values clinically have been developed for the prognosis and diagnosis of HNSCC [11–14]. However, the clinical utility and reproducibility of these models are uncertain [15]. The modified proteome represents the final result of different molecular pathways and has the potential for the therapeutic targeting of malignancies. However, due to the complex regulatory processes occurring after mRNA is transcribed, the abundance of proteins in a cell can never be fully predicted or explained by their corresponding mRNA expression [16]. As such, proteomic analysis of tumors can provide researchers with large amounts of bioinformatics data different from that obtained by RNA or DNA sequencing.

In recent years, protein-based prognostic signature models have been developed to predict cancer survival. For example, Xie et al. [17] developed a 3-protien predictive risk score model for high-grade serous ovarian cancer's progression-free survival (PFS) and overall survival (OS). Han et al. [18] identified 4 protein biomarkers that are prognostic for kidney renal clear cell carcinoma. Patil and Mahalingam [19] successfully predicted lower-grade glioma patients' survival using a 4-protein prognostic signature.

The Cancer Proteome Atlas (TCPA) is an open-access bioinformatics resource that belongs to The Cancer Genome Atlas (TCGA) Project [20, 21]. It contains protein expression data of many tumor cell lines formed by reverse-phase protein arrays (RPPAs) [20, 21]. In this paper, a novel protein signature was constructed and checked for determining the prognosis of HNSCC patients using the functional proteomic data collected from TCPA.

## 2. Material and Methods

### 2.1. Patients and Proteomic Data

The functional proteomic data of 347 HNSCC patients were obtained from TCPA online database (http://tcpaportal.org), and TCGA (https://cancergenome.nih.gov/) provided corresponding clinical and follow-up data. Upon removing fragmentary clinical follow-up records, this article enrolled the data of 332 cases.

The 332 patients were grouped randomly as training set (*n* = 168) and test set (*n* = 164), with the aim of comparability of variables in the 2 sets. The prognostic model was developed using the training set and verified via the test set.

### 2.2. Survival Analysis Based on the Functional Proteomic Data in TCPA Database

Candidate proteins were selected from the functional proteomic data using the Kaplan-Meier method and univariate Cox proportional hazards regression analysis in the survival R package software version 3.6.3. First, the univariate Cox regression analysis was performed for the associations between patient OS and protein expression. Next, we repeatedly classified the 168 patients in the training set into low or high expression on the basis that the protein expression identification was < median (low) or > median (high). Both groups were kept the same patients in number. The median level was determined by the number of patients in both groups. Survival differences between the low- and high-expression groups were examined with the 2-sided log-rank test. Only proteins with a value of *P* < 0.05 were considered candidate proteins.

### 2.3. Definition of Protein-Related Prognostic Model and Risk Score

Based on the above method, 7 proteins were chosen to be candidates and received a multivariate Cox regression analysis to identify the preferred mathematical model with the Akaike Information Criterion (AIC). A predictive model by AIC has the best informative efficacy and goodness of fit. After the multivariate Cox regression analysis, the risk score of each patient was calculated by a formula: Survival Risk Score = ∑_*k*=1_^*n*^(*C*_*k*_ × *V*_*k*_). Specifically, *n* is prognostic proteins' number; *C*_*K*_ is the *K*th protein's coefficient in the multivariate Cox regression analysis; and *V*_*k*_ represents the *K*th protein expression value. Proteins were considered to have a high-risk signature (*C*_*K*_ > 0) and a low-risk signature (*C*_*K*_ < 0). All functional proteomic data were analyzed using the R package software version 3.6.3.

### 2.4. Risk Stratification and Survival Curve

Based on the calculated risk score, the 168 patients were pigeonholed as low-risk (< median score) and high-risk (> median score) groups. With the Kaplan-Meier method and R software, an OS curve was generated. And the survival time differences were compared by the log-rank test.

We also developed 3 survival curves of the low- and high-expression groups that were based on the final 3 proteins included in the predictive model. Finally, risk curves, survival maps, and heat maps were plotted to show the risk score's distributions of each protein for training set patients.

### 2.5. Independent Analysis of Prognosis and Comparison of Receiver Operating Characteristic (ROC) Curves

To appraise clinical factors' prognostic ability (age, gender, disease stage, and smoking history) and the risk score, the multivariate and univariate Cox regression analyses were conducted using survival state and time as the dependent variables; and *P* < 0.05 was considered that the factors had independent prognostic values.

Besides, the ROC curve analysis was employed for evaluating the performance of the prognostic model and the clinical parameters, and the R Survival ROC package was used for drawing and analyzing the ROC curve. The calculation of areas under the ROC curves (AUCs) was gone on for comparing the prognostic value of clinical factors and the prognostic model.

### 2.6. Validation in the Testing Set and in Combined Cohorts

Based on the results obtained with the training set, we calculated the 164 patients' risk scores in the test set. The subjects were partitioned as low- and high-risk groups in the light of the median score. In addition, this process was also carried out in all 332 patients combined (combined cohort). The Kaplan-Meier survival curves of the testing set and that of the combined testing and training set were plotted, and survival differences between the low- and high-risk groups were compared via the log-rank test. And the model's prognostic value was estimated by the AUC of both ROC curves.

### 2.7. Protein Coexpression Analysis and the Sankey Diagram

To identify the potential proteins correlated with the 3 proteins in the model, proteins identified in the functional proteomic data whose expressions were significantly correlated with the proteins in the predictive model were identified using 2-sided Pearson's correlation coefficient analysis and the *Z*-test. Proteins with an absolute Pearson's correlation coefficient value of >0.4 and *P* value < 0.001 were considered to have positive or negative correlation with the 3 proteins in the prognostic model. A Sankey diagram was plotted using the “ggalluvial” R software package to illustrate the potential correlations of the proteins.

## 3. Results

### 3.1. Patient Characteristics

Table 1 presents 332 HNSCC cases' data clinically in the testing (*n* = 164) and training (*n* = 168) sets. In these cases, 200 suffered Stage IV, 61 Stage III, 57 Stage II, and 14 Stage I disease. Patients were randomly divided into the testing set (*n* = 164) and training set (*n* = 168). Few obvious differences were observed in variables clinically (e.g., age, gender, TNM stage, survival time, and survival status) between the two sets (all, *P* > 0.05) (Table 1).

### 3.2. 7 Proteins Were Selected as Candidate Proteins to Construct a Prognostic Model

A total of 237 proteins were screened for the functional proteomic data of HNSCC from TCPA datasets. As shown in Figure 1 (volcano plot), there were 8 proteins that were defined as low risk and 16 proteins that were defined as high risk. The 24 proteins' prognostic values were determined via the univariate Cox regression analysis (all, *P* < 0.05). Then we conducted the Kaplan-Meier analysis, and 7 proteins were selected as candidate proteins to build a prognostic model (Table 2).

### 3.3. The 3-Protein Signature Constructed from X4EBP1_pT37T46, HER3_pY1289, and NF2 Was Established by the Multivariate Cox Regression Analysis

A 3-protein prognostic model was established by 3 of the 7 proteins selected with the stepwise multivariate Cox regression analysis. The 3 proteins selected were X4EBP1_pT37T46, HER3_pY1289, and NF2. The predictive model was based on the summed expressions of the 3 proteins weighted by their relative coefficients. The relative coefficients were calculated using the multivariate Cox regression and represented each protein's risk degree (Table 3). The multivariate survival analysis outcomes using the 3 proteins are shown in Figure 2.

Every patient's survival risk score was calculated through the formula: Survival Risk Score = (−0.544877895 × X4EBP1_pT37T46 expression value) + (1.016464597 × HER3_pY1289 expression value) + (1.122403466 × NF2 expression value). Of the 3 proteins, the coefficient of X4EBP1_pT37T46 was negative in the Cox regression analysis indicating it is protective since high expression is associated with longer OS. Conversely, the coefficients of the other 2 proteins (HER3_pY1289 and NF2) were positive and thus were considered risk factors because higher expression of the 2 proteins meant shorter OS.

### 3.4. The 3-Protein Signature Can Predict the Survival of HNSCC Patients

First, 3 survival curves of the high- and low-expression groups on basis of the expression of the 3 proteins in the predictive model were developed (Figures 3(a)–3(c)). The Kaplan-Meier survival curves of the 2 groups based on the 3 proteins' expression were significantly different (*P* value, log-rank test).

Next, with the median risk score described previously as a standard, training set's patients were divided into a high-risk group and a low-risk group. Survival analysis indicated a great difference in the high- and low-risk groups' survival time, further confirming the prognostic effectiveness of the 3-protein signature (Figure 3(d)). The risk curve, survival map, and heat map of the 3-protein signature are shown in Figure 4. As shown in Figures 4(a)–4(b), the deaths in the high-risk areas were obviously larger than those in the low-risk areas. As shown in Figure 5(c), the expression patterns of the 3 proteins were correlated with risk scores.

### 3.5. The 3-Protein Signature Have Better Prognostic Value than Clinical Factors

Figures 5(a)–5(b) exhibit the results of the univariate and multivariate Cox regression analyses of the 3-protein signature and clinical factors. The OS had significant association with the risk score and N stage, and the 3-protein signature risk score and N stage were both independent predictors of survival. To compare the 3-protein signature risk score and the clinical factors' prognostic power, ROC curves of each independent variable were plotted, and the AUCs were calculated (Figure 6). The results showed greater AUC of the 3-protein signature (0.750) than the AUC of N stage (0.624) in the training set, indicating that the 3-protein signature exhibited better sensitivity and specificity in predicting survival. Taken together, these results indicate that the 3-protein signature exhibits better predictive value for survival of HNSCC cases (hazard ratio (HR) = 1.471, 95% confidence interval (CI): 1.255-1.726, *P* < 0.0001, Figure 5(b)), as compared with conventional clinical factors like age, sex, smoking history, and TNM stage.

### 3.6. The 3-Protein Prognostic Signature Model Exhibits Good Performance in the Testing Set

The Kaplan-Meier survival curves and ROC curves of the 3 proteins in the testing set and combined cohort set are shown in Figures 7(a)–7(d). Consistent with results of the training set, differences (*P* < 0.05) of OS were statistically significant between the low- and the high-risk groups in the testing set and combine cohort. The AUC for the 3-protein signature in the testing set was 0.655 (Figure 7(b)) and in the combined cohort was 0.699 (Figure 7(d)), suggesting good performance of the 3-protein signature for predicting OS.

### 3.7. Other Proteins Potentially Correlated with the Survival of HNSCC

Applying Pearson's correlation and the *Z*-test to the 3 proteins in the model and other proteins identified showed that there was coexpression between 12 proteins and 1 of the 3 proteins in the model (∣Pearson correlation coefficient | >0.4 and *P* < 0.001). The Sankey diagram showing the correlations of the proteins is shown in Figure 8. Thus, the 12 proteins may be related to HNSCC's prognosis.

## 4. Discussion

In this study we identified 3 proteins (X4EBP1_pT37T46, HER3_pY1289, and NF2) related to HNSCC patients' survival and developed a model using the 3 proteins for predicting their OS. A training set was used to develop the model, and the model was validated with a testing set. The AUC for the 3-protein signature in the testing set was 0.655 and in the combined cohort was 0.699, indicating great performance of the 3-protein signature in the OS prediction of HNSCC patients. In addition, the 3-protein signature exhibited better predictive value for survival of HNSCC patients as compared with conventional clinical factors (age, sex, smoking history, and TNM stage).

HNSCC is a relatively common malignancy and is very common in certain parts of the world [22]. Although there have been many advances in understanding of the molecular biology of HNSCC [1, 4, 7–9], as well as treatment options, the mortality of patients with HNSCC remains high. As such, there is a need for the development of novel markers to predict prognosis and help guide treatment.

Bioinformatics studies have screened molecular biomarkers such as mRNA, miRNA, and lncRNA to predict the prognosis for HNSCC patients [11, 12, 23]. Advances in high-throughput proteomics techniques allow the quantitative assessment of large numbers of proteins in multiple specimens. As an antibody-based protein microarray dot-blot platform, the reverse-phase protein array (RPPA) allows a large number of biological samples' quantitative measurement in protein expression level simultaneously as antibodies with high quality are available [24–26]. Many studies have used the RPPA technique to study protein biomarkers relevant to cancer progression, treatment selection, and prognostic prediction [19, 27].

With major advances in bioinformatics, proteomics, and techniques of gene analysis, a great deal of researchers has contributed themselves to developing signatures using different methods for predicting the prognosis of patients with head and neck cancer. Prognostic signatures have been developed using miRNA [28, 29], alternative splicing [30], immune function molecules [31], and a signature according to m^6^A RNA methylation regulators [32].

In a study similar to ours, Zhao et al. [33] reported a 5-protein signature for predicting HNSCC prognosis. Notably, the OS was much worse in patients with high-risk scores than that in those with low-risk scores in the subgroups of male sex, tumor grade 1-2, age < 60 years, and disease Stages III-IV. OS differences were not significant in patients in the subgroups of female sex, age ≥ 60 years, tumor grade 3-4, and disease Stages I-II. In other notable research, Jin et al. [34] reported that p53-targeted lncRNA-p21 serves as a tumor suppressor through suppressing JAK2/STAT3 signaling pathways in HNSCC. Zhang et al. [14] developed a model using 5 genes as a novel signature for the prognosis prediction of people with laryngeal cancer (KLHDC7B, MMP1, DPY19L2P1, HOXB9, and EMP1). The ROC curve analysis suggested good effect of the 5-gene signature on predicting laryngeal cancer prognosis (AUC = 0.862, *P* < 0.05). Guo et al. [23] reported a 6-mRNA (ZNF324B, YIPF4, TMC8, PDGFA, PCMT1, and FRMD5) signature model for determining HNSCC prognosis. The AUC of the model for predicting OS was 0.745 (*P* < 0.001). Wang et al. [35] recently reported that 3 microRNAs (has-miR-1911, has-miR-499a, and has-miR-99a) were independent risk factors significantly related to patients with head and neck cancer in survival (all, *P* < 0.01). In addition, GO and KEGG analyses presented the association of cancer prognosis with the JAK STAT signaling pathway and certain metabolic pathways. In a unique study, You et al. [36] used cDNA microarrays and bioinformatics methods to study radio-resistance in head and neck carcinoma and identified 4 key functional pathways and molecular markers that greatly promoted radio-resistance. A recent report by Ribeiro et al. [37] studied tumor specimens of 40 patients with HNSCC undergoing tumor resection, and tumor-adjacent tissues from 32 of the patients. The authors identified a proteomic signature based on 3 proteins (DHB12, HMGB3, and COBA1) and developed a model that included the 3 proteins and tumor stage that exhibited >80% predictive accuracy for the development of metastasis and recurrence.

This study's primary demerit is that the analysis was based on information contained in large databases. While this method provides important information and we were able to develop a protein signature predictive of the OS of patients with HNSCC, clinical validation of the results was not performed. Clinical validation of the results was not part of the research design and hence was not performed. While the results are compelling, they need to be verified through clinical study of HNSCC patients.

## 5. Conclusion

In this report, we developed a 3-protein signature to predict HNSCC patients' survival. The AUC for the 3-protein signature in the testing set was 0.655 and in the combined cohort was 0.699, indicating the favorable role of the 3-protein signature in HNSCC patients' OS prediction. In addition, the 3-protein signature exhibits better predictive value for survival of HNSCC patients as compared with conventional clinical factors like gender, smoking history, age, and TNM stage. These results add relevant information to the medical literature to help guide the management of patients with HNSCC.

## Figures and Tables

**Figure 1:** Volcano plot of the 24 prognosis associated proteins. Green dots represented low-risk proteins; red dots represented high-risk proteins (*P* value filter = 0.05). HNSCC: head and neck squamous cell carcinoma. The figure was created with the R package software version 3.6.3, the R Foundation.

**Figure 2:** Forest plot of the 3-protein signature. A hazard ratio (HR) < 1 meant protective (i.e., X4EBP1_pT37T46), and HR > 1 suggested increased risk (i.e., HER3_pY1289 and NF2). The multivariate survival analysis revealed the 3 proteins were independent prognostic factors. The figure was created with the R package software version 3.6.3, the R Foundation.

**Figure 3:** Kaplan-Meier (KM) curves of the 3 proteins in the training set. The shaded area stood for the 95% confidence interval (CI) of the curves. (a) KM survival curves of 168 persons with HNSCC partitioned as high-expression and low-expression groups by X4EBP1_pT37T46. (b) KM survival curves for NF2. (c) KM survival curves for HER3_pY1289. (d) Survival analysis in survival time of the high- and low-risk groups. *P* values were derived from the log-rank test. The figure was created via the R package software version 3.6.3, the R Foundation.

**Figure 4:** The distribution of risk scores and the expression heat map of the 3 proteins. Red dots were high-risk patients, and green dots were low-risk patients. (a) Risk curve of 168 HNSCC patients arranged in order. (b) Survival status map. (c) Expression heat map of the 3 prognostic proteins. The figure was made through the R package software version 3.6.3, the R Foundation. HNSCC: head and neck squamous cell carcinoma.

**Figure 5:** Forest plots derived from (a) univariate and (b) multivariate Cox regression analyses. The risk score and N stage (both, *P* < 0.05) were considered independent predictors. The figure was constructed by the R package software version 3.6.3, the R Foundation.

**Figure 6:** Conventional clinical factors and receiver operating characteristic (ROC) curves for the 3-protein signature in the training set. The area under the ROC curve (AUC) of protein model was 0.750, which was greater than that of other factors. The figure was established using the R package software version 3.6.3, the R Foundation.

**Figure 7:** Kaplan-Meier and receiver operating characteristics (ROC) curves for the 3-protein signature in both validation sets. The shaded area in Kaplan-Meier curves meant the 95% confidence interval (CI) of the curves. The risk table under the survival curve suggested the number of patients remaining at each time point. (a) Kaplan-Meier curves for the 3-protein signature in the test set. (b) ROC curves for the 3-protein signature in the test set. (c) Kaplan-Meier curves for the 3-protein signature in the combined cohort. (d) ROC curves for the 3-protein signature in the combined cohort. *P* values derived from the log-rank test. The figure was created with the R package software version 3.6.3, the R Foundation.

**Figure 8:** The Sankey diagram of the coexpression between 12 correlated proteins and 1 of the 3 proteins in the model. The figure was built via the R package software version 3.6.3, the R Foundation.

**Table 1:** Clinical data of patients in the training set and testing set.

Variates	Total (*n* = 332)	Training set (*n* = 168)	Testing set (*n* = 168)	*P* value	Method
Age, years	60.98 ± 12.21	60.39 ± 12.60	61.57 ± 11.82	0.379	*t* test
Gender					
Female	93 (28.01%)	50 (29.76%)	43 (26.22%)	0.472	*χ* ^2^ test
Male	239 (71.99%)	118 (70.24%)	121 (73.78%)		
Stage					
I	14 (4.22%)	8 (4.76%)	6 (3.66%)	0.112	*χ* ^2^ test
II	57 (17.17%)	35 (20.83%)	22 (13.41%)		
III	61 (18.37%)	24 (14.29%)	37 (22.56%)		
IV	200 (60.24%)	101 (60.12%)	99 (60.37%)		
T stage					
1	23 (6.93%)	10 (5.95%)	13 (7.93%)	0.070	*χ* ^2^ test
2	99 (29.82%)	61 (36.31%)	38 (23.17%)		
3	83 (25.00%)	37 (22.02%)	46 (28.05%)		
4	127 (38.25%)	60 (35.71%)	67 (40.85%)		
N stage					
0	150 (45.18%)	75 (44.64%)	75 (45.73%)	0.472	Fisher's exact test
1	44 (13.25%)	18 (10.71%)	26 (15.85%)		
2	131 (39.46%)	71 (42.26%)	60 (36.59%)		
3	7 (2.11%)	4 (2.38%)	3 (1.83%)		
M stage					
0	330 (99.40%)	167 (99.40%)	163 (99.39%)	0.745	Fisher's exact test
1	2 (0.60%)	1 (0.60%)	1 (0.61%)		
Smoking history					
Nonsmoker	124 (37.35%)	62 (36.90%)	62 (37.80%)	0.865	*χ* ^2^ test
Smoker	208 (62.65%)	106 (63.10%)	102 (62.20%)		
Survival time (mean), units	1.83 ± 2.63	1.83 ± 2.32	2.01 ± 2.92	0.523	*t* test
Survival status					
Alive	203 (61.14%)	104 (61.90%)	99 (60.37%)	0.774	*χ* ^2^ test
Dead	129 (38.86%)	64 (38.10%)	65 (39.63%)		

Survival time and age presented as mean ± standard deviation and other data as count (percentage).

**Table 2:** Seven proteins identified by the Kaplan-Meier analysis to construct a prognostic model.

Protein	*P* value^a^	HR	95% CI (lower)	95% CI (upper)	*P* value^b^
X4EBP1_pT37T46	0.01899	0.577475	0.39181	0.85112	0.005528669
BAK	0.034163	1.449073	1.067948	1.966213	0.017211745
EGFR_pY1173	0.048016	1.240488	1.021306	1.506709	0.02981831
HER3_pY1289	0.009158	3.574414	1.405492	9.090362	0.007479537
NF2	0.00516	3.409989	1.589803	7.314126	0.001628719
BRAF_pS445	0.029428	0.129952	0.039403	0.428582	0.000803566
KEAP1	0.035003	0.630596	0.406964	0.977117	0.039059154

CI: confidence interval; HR: hazard ratio. ^a^*P* value derived from the Kaplan-Meier method. ^b^*P* value derived from the univariate Cox regression analysis.

**Table 3:** Risk degree of the 3 proteins included in the model.

Protein	Coefficient	HR	95% CI (lower)	95% CI (upper)	*P* value
X4EBP1_pT37T46	-0.544877895	0.579913	0.397571	0.845882	0.00467
HER3_pY1289	1.016464597	2.763408	1.055127	7.237447	0.038527
NF2	1.122403466	3.072229	1.419427	6.649579	0.004385

CI: confidence interval; HR: hazard ratio. *P* values derived from the univariate Cox regression analysis.

## Data Availability

The data used to support the findings of this study are available from the corresponding author upon request.
